# Personal Competition Among Sports Players and Their Performance as a Team: A Moderated Mediation Model

**DOI:** 10.3389/fpsyg.2022.862599

**Published:** 2022-03-28

**Authors:** Jinling Li

**Affiliations:** School of Public Education, Shandong College of Arts, Jinan, China

**Keywords:** personal competition, playing dumb, team performance, task interdependence, knowledge hiding behavior

## Abstract

Personal competition among colleagues and co-workers has been observed in order to prove their professional superiority over others. Such behaviors have grave consequences on the overall team performance. The aim of this study was to investigate the role of personal competition on team performance incorporating the mediating role of the playing dumb behavior of knowledge hiding. The study has further checked the moderating effect of task interdependence on the relationship between personal competition and playing dumb. Data for the present study had been collected through questionnaires from the sports players actively associated with games through their educational institutes in China. The sample size of the study was 339, selected on the basis of convenience sampling. Smart PLS had been employed to analyze the data through structural equation modeling (SEM). The results of the study showed a strong impact of personal competition on team performance and the playing dumb variable. Furthermore, playing dumb has been found to have a strong mediating impact on team performance. The study has theoretically contributed to the literature of competition and performance by investigating the mediating role of playing dumb. The study also offers certain practical implications to the managers of the corporate world to devise such human resource policies that take appraisals from the colleagues so as to rectify the negative workplace behaviors and could be worked out accordingly.

## Introduction

Growing international competition, as well as the demand for different talents, knowledge, and creativity fueled the growth of collaborative work structured in teams as basic organizational building blocks that need faster and more flexible reactions. Among the most prevalent developments in complicated and dynamic work settings is the implementation and utilization of various types of teams (Ghosh et al., 2018; Zaccaro et al., 2020). Complex challenges necessitate the collaborative creation of inventive solutions, as well as the building of collaboration connections that offer employees the inspiration, knowledge, resources, and support they need to create, market, and implement their new ideas (Perry-Smith and Shalley, 2003). Therefore in this scenario, teams have emerged as a critical component of organizational success and global knowledge generation, because they’re more inclined than individual people to create higher returns, find novel solutions, and therefore improve performance (Edmondson and Harvey, 2018; O’Neill and Salas, 2018).

Performance is characterized as a sequence of activities that produce a scale for achieving corporate goals (Motowidlo and Kell, 2012). Studies on team performance have advanced dramatically in distinguishing between team performance and effectiveness in recent times. A link between a team’s performance and the activities they conduct while completing a job, as well as the link between the effectiveness and the measurement of the outcomes of these operations, had significant effects (Salas et al., 2009). Initially, forecasting team performance indicators linked to a diverse collection of behaviors have an impact on the work teams’ operations. Team performance is defined as the total of positive anticipated behaviors associated to promoting teamwork and social performing change over a period of time in this method (Motowidlo and Kell, 2012). Furthermore, performance and efficiency assessments are assessed by comparing statistics with suitable behavior explanations (Wildman et al., 2013). To strengthen the assessment process and appropriately grasp the multifaceted character of team performance, both aspects require a filter of explanatory factors (Salas et al., 2017).

In sports, the contrast between the team and individual players is crucial. Since over seven decades of research, very little is understood regarding inter-personal distinctions among individuals and team athletes. Researchers found that team players are more extroverted and less conscientious than solo athletes in their assessment of the relationship between sports and personality (Allen et al., 2011, 2013). In terms of social skills, no apparent differences were discovered (Landkammer et al., 2019). We assume that the lack of a link between athletics affiliation with social skills is due to previous studies focusing on general skills and personality traits. People who participate in team sports usually train alongside other sportsmen. This seems to be true not only for team sports but also for individual ones. As a result, when sportsmen are preparing for tournaments or competitions, they are generally in social settings (Evans et al., 2012; Martin et al., 2014). Furthermore, while playing as a team against other teams, such as during soccer games or relay swimming contests, athletes rely on one another since they are positively interdependent.

Competition or adverse dependency among sportsmen or teams is, in reality, a key feature of the social environment of professional team sports. Competing individuals seldom cooperate with one another during a competitive circumstance since doing so would jeopardize their chances of success. Pure competition, on the other hand, is uncommon in real-life social situations (Johnson et al., 1981; Esses et al., 1998). Sports tournaments, for example, need at least a basic level of collaboration between competitors in the application of basic standards. People may be forced to compete and collaborate with the same participants in particular situations. This is a social situation characterized by the so-called mixed-motive interdependence in psychological terminology. Furthermore, unlike the mixed-motive interdependence literature’s typical social dilemmas, co-opetition somehow doesn’t allow one to choose between competing and collaborating (Landkammer and Sassenberg, 2016).

Even with all these parallels among team and individual sports mentioned previously, team sports are intrinsically more competitive. On the one extreme, team players are always competing against their colleagues (e.g., for starting roles and other status-related resources). Officials or coaches also could try to encourage such intra-team games in the hopes of improving their athletes’ performance. Team players must work together with their colleagues throughout the team performance to complete the objective, progress as a team, and succeed against the other squads. Cooperation in this context entails not just working toward a common objective, but also demonstrating behavioral interdependence by demonstrating conduct that helps other athletes do better (Landkammer et al., 2019). Individual sports have a lower demand for simultaneous competition and cooperation while trying to perform. Individual players must engage cooperatively in general, in order to work effectively with their support staff in top sport, although cooperative conduct while performing is less necessary than in team sports.

Individual sports, frequently demand athletes to surpass others during practice or competitions. Individual results are accumulated to a team performance in baton contests (e.g., swimming), but no collaborative activity inside the team is necessary throughout the race (Landkammer et al., 2019). Competitiveness among team members, in particular, has a detrimental influence on the sharing of task-relevant knowledge. Individuals vying for a greater position, attempting to optimize their personal results, and striving to be the first to know the correct option that has all demonstration for this (Sassenberg et al., 2007; Toma and Butera, 2009; Steinel et al., 2010; Ray et al., 2013; Toma et al., 2013). These effects can be explained on a cognitive level by a depiction of competition which eliminates or restricts collaborative thinking and behavior: individuals depend on this representation when encoding a situation as competitive, and they stop cooperating and behaving in a competitive manner. To put it another way, competition should naturally limit cooperative thinking and conduct (Landkammer and Sassenberg, 2016).

A lot of research has been conducted on knowledge sharing perspectives in positive team performances and organizational success in the past. Knowledge hiding behaviors are relatively new entrants in this setup of organizations. Connelly et al. (2012) initially reported that there are three types of knowledge hiding, namely, playing dumb, rationalized knowledge hiding, and evasive hiding. These are the behavioral aspects of knowledge hiding which are associated with different setups of organizations and individuals. Several types of research like Fong et al. (2018) have been conducted in order to evaluate the impact of knowledge hiding on team creativity and evaluated the contingent role of task interdependence between knowledge hiding and team creativity. These results indicated that there was a significant impact of knowledge hiding on the creativity of the teams which is the antecedent of team performance.

This kind of relationship hinted about exploring the specific type of knowledge hiding, i.e., playing dumb in the context of sports psychology while evaluating the role of personal competition on team performance. So, this gap provided the basis for modeling the current research. In this context, the mediation of the playing dumb perspective of knowledge hiding behavior was not studied before. So, playing dumb was conceptualized as a mediator between personal competition and team performance. Another gap was found in this research that task interdependence was utilized as a moderator between knowledge hiding and team creativity while moderation between personal competition and knowledge hiding was not explored. This also hinted toward its possible moderating effect between personal competition and the mediator of our research. Several types of research focused on the competitive aspect of sportsmen toward team performance such as Landkammer and Sassenberg (2016), but they did not evaluate the impact of components of this competition such as personal competition on team performance. This hinted at us for evaluating the impact of personal competition on team performance.

These gaps in the previous research posed some questions such as “does personal competition have any role on the performance of the team?” If there is any impact of personal competition among the sportsmen or teammates then what factors could regulate or mediate the function of such a relationship? As playing dumb is a kind of knowledge hiding, and knowledge hiding hinders team performance, how could playing dumb affect the relationship between personal competition and team performance? Another question was raised that how task interdependence could regulate the relationship of personal competition with mediating playing dumb? To answer these questions, this research was designed with several objectives such as exploring the relationship of personal competition with team performance, addressing the mediating role of playing dumb between personal competition and team performance, and evaluating the moderating mediated impact of task interdependence on knowledge hiding leading to team performance.

## Theoretical Support and Hypothesis Development

Social comparison theory is one of the more well-known viewpoints on the competitiveness/situation relationship. Unlike social interdependence theory, when rivalry is fundamentally established, social comparison theory competition is driven by either a person’s need for honest self-evaluations about personal talents in an attempt to discover areas for improvement (Festinger, 1954). Competition is just a comparison activity by definition, as it serves as a measure of one’s talents in relation to someone or himself. If there’s not an impartial, measurable outcome through which one may assess their ability, competition serves as such evaluation. Competition aids in negotiating difficult goal attainment settings in which there are seldom objective, discernible criteria as long as the comparative other is similarly capable. In general, social comparison theory research on competitiveness finds three variables that promote comparative considerations and, as a result, competitive nature (Festinger, 1954). Initially, whenever performing a task that is essential to one’s consciousness, competing social comparisons become much more prominent, resulting in enhanced effort and commitment (Tesser, 1988; Garcia et al., 2013). Overall, the value of the contrast to a team’s or person’s self-construal is increased by the task’s priority, leading to more effort in pursuit of higher performance.

Moreover, while the other will have the same qualities, level of skill, and characteristics as the other, such as sexual identity, ethnicity, nationality, and economic status, the contrast is very striking (Dakin and Arrowood, 1981; Kilduff et al., 2010). The comparison has more weight if the comparative other is similar in form or function (Festinger, 1954). The last criteria concern the player’s degree of affective proximity to the aim. When it comes to people who are close to you, including a colleague or a brother, comparisons are more powerful (Tesser, 1988). People on the spectrum provide less helpful hints to friends than strangers, are more intimidated by a friend’s achievement than a stranger’s, and function effectively (Zuckerman and Jost, 2001; Locke, 2007). In one study, scientists found that when competitors could identify their counterparts in three studies, they lasted longer and did better than when the contemporaries were unidentified (Haran and Ritov, 2014). Whenever individuals self-identify within their community and get self-evaluative knowledge through intergroup comparisons rather than personal comparisons, a similar comparison process occurs. Team members may rely on performance comparisons as assessment tools in multilevel social circumstances where contextual signals regarding performance are lacking (Ding et al., 2018).

According to the social identity theory, comparing groups enhances in-group bias, thus when teammates compete, they evaluate team strengths while simultaneously erecting barriers here between and out-group (Brown, 2000). The above appears to have significant consequences for the impact of competition on the settlement of the intergroup conflict. Teams that compete compare themselves to one another, which can lead to the formation of organizational silos defined by a we-vs-them mindset. Based on these inferences, we evaluated the personal competition for team performance. The action regulation theory describes the ways people govern their objective conduct *via* many activities or procedures, including goal formation, externally and internally orientation, preparation, implementation, and assessment. Work planning, cooperation in tasks (i.e., collaboration and knowledge exchange), work evaluation (procedures and quality assurance) (Frese and Zapf, 1994; Tschan, 2002; Rousseau et al., 2006), and adaptation behaviors are all behaviors that assure team performance (such as backing-up, coaching, problem-solving, and team innovative behavior) (Rousseau et al., 2006; Granåsen, 2019).

Despite the fact that Rousseau’s model is one of the most effective measures of generic collaboration, in-depth specification is required to adapt it to various real-world settings (Ficapal-Cusí et al., 2021). The formation of ideas in the team’s creative powers, according to the Social Cognitive Theory, stimulates the team’s collaborative behavior. The combination of collective efficacy and creative self-efficacy produces creative collective efficacy (Bandura et al., 1999; Morgeson and Hofmann, 1999). It is a person’s conviction in a group’s ability to achieve innovative solutions. A group’s creative performance was found to be enhanced by creative collective efficacy (Morgeson and Hofmann, 1999; Tierney and Farmer, 2002; Luthans et al., 2007; Shin and Zhou, 2007; Cheng and Yang, 2011; Salanova et al., 2014). Team members are more likely to integrate, share, or restructure their ideas into something new if they have strong shared views about their team’s creativity (Shin and Zhou, 2007). These theories provided a basis for checking the impact of personal competition on team performance.

### Personal Competition and Team Performance

Competitiveness, also known as innate competition or deliberate competitiveness, is an individual difference that results in a propensity for competition. Competition may be beneficial, defined by increased drive and involvement, or harmful, characterized by suspicion and intense negative feelings, dependent on how it develops (Kohn, 1986; Ryckman et al., 1990; Johnson and Johnson, 1991; Murayama and Elliot, 2012). The two broad conditions were expanded to three distinct competitive tendencies by personality scientists, i.e., competition avoidant, hypercompetitive, and personal growth (Ryckman et al., 2009). Horney describes the second type of neurotic competitiveness as competition avoidance. This attitude stems from being afraid of ruining others’ admiration and acceptance, either through winning the competition (leading in anger from the loser) or failing in the competition (resulting in resentment from the loser). Ignoring persons shun competition as possible in order to prevent a decrease in personality (Horney, 1937; Ryckman et al., 2009). Whenever they can’t get away from that too, the competitive avoidant destroys their own prospects of success. They do so by participating in a range of behaviors such as mocking themselves, downgrading their own intelligence and aptitude, and engaging in distracting activities that purposely distract them from the competition as an excuse.

Personal development competitiveness is the final of the three orientations, and it views competition as a type of personal growth and development, self-discovery, and consciousness. Personal competition, on the other hand, is a healthy sort of individual competitive behavior in which participants focus on “the enjoyment and mastery of the work” rather than on succeeding. A personal competition exhibits a high degree of self, success, connection, compassion for others’ well-being, and forgiveness, as well as lower levels has dominant behaviors, violence, and psychopathy. Unlike unhealthy kinds of competition, this attitude represents a healthy and constructive sort of competition (Ryckman and Hamel, 1992; Ryckman et al., 1996, 1997; Collier et al., 2010). Though contextual competitiveness and individual competitiveness are well-known, competition appears to be a communal construct as well. Several, widely obtainable examples of a team’s sustained competitiveness resulting in collective goal attainment may be found in personal anecdotes.

Collaborative competitiveness emerges out of a bottom-up emergent process in which lower-level constructs converge through social contact, trade, and combinations to generate a higher-level emerging attribute of the team, to borrow the terminology from Klein and Kozlowski (2000) and Garcia and Tor (2009). We describe collective competitiveness as a team’s competitive performance that results in a preference for competition, similar to how individual competitiveness is defined. This results from team members’ interactions in which they come to an agreement on their common competitive impulses (Chan, 1998). As team members connect with each other, people transmit meaning drawn from their own competitive personalities, which allows them to communicate their viewpoints on the surroundings. They define the competitive situation for one another over time as they share until an emerging form of competition emerges and the group comes to understand goal interrelations in the same way (Fulmer and Ostroff, 2016; Swab and Johnson, 2019). Based on these arguments, we developed the following hypothesis.

**H_1_**. Personal competition has an effect on team performance.

### Personal Competition, Playing Dumb, and Team Performance

According to Connelly et al. (2012), playing dumb is the constituent or type of knowledge hiding in which a person (player in our context) hides the information from the colleagues (team players) for certain reasons. Playing dumb, in our context, refers to the hiding of information from others due to competition with other players. It could be understood that personal competition leads to accomplishing certain tasks and due to achievement sense, negative behavior sometimes develops at a personal level. The impact of personal competition could lead to the development of knowledge hiding or playing dumb specifically. Similarly, this negative behavior leads to the deteriorated performance of the team in return. Certain research in the past has evaluated the impact of knowledge hiding on team performance in terms of creativity such as Fong et al. (2018) but did not evaluate the role of personal competition on playing dumb which is a type of knowledge hiding.

Team performance is determined by the amount and quality of work performed by a team and is the result of all team members’ combined efforts. Team members should be able to enable team processes such as coordination and communication in order to guide, coordinate, and evaluate teamwork to improve team performance. Teamwork procedures may be harmed if team members intentionally hide knowledge from their coworkers, which may result in poor team performance. Knowledge concealment may cause a change in attention from a team to a more narrow and personal focus, obstructing staff coordination and communication and lowering team performance (Burke et al., 2006). To overcome this gap, we devised the following hypotheses for evaluation of the impact of personal competition on knowledge hiding and the impact of knowledge hiding (playing dumb) on team performance.

**H_2_**. Personal competition has an effect on playing dumb perspective of knowledge hiding.

**H_3_**. Playing dumb has an effect on team performance.

Certain studies have also evaluated the mediating role of playing dumb in various perspectives, i.e., interpersonal conflict and psychological strain (Venz and Nesher Shoshan, 2021), territorial feeling, and innovation of employees (Guo et al., 2022), etc. Several researchers have focused on mediating the role of knowledge hiding in different perspectives, i.e., abusive supervision and employee creativity (Jahanzeb et al., 2019). Based on this analogy, we hypothesized that playing dumb would mediate the process of team performance due to personal competition.

**H_4_**. Playing dumb mediates the relationship between personal competition and team performance.

### Task Interdependence as a Moderator

Interdependence between tasks promotes communication and collaboration, as well as mutual adaptation between acquirers and targets. In the literature on knowledge management, such a task feature has been recognized as a contextual moderator. When tasks are interdependent from other team members, the relationship between personal competition and knowledge hiding should be less negative (Bachrach et al., 2006; Staples and Webster, 2008). On the one hand, task interdependence as a moderator represents an unproven aspect of the original knowledge-hiding theory (Černe et al., 2014). Thus, the negative effects of knowledge hiding could be mitigated in an environment relating to information exchange and collaboration. Because it highlights the necessity of joint effort and collaboration among team members, task interdependence appears to reflect such a climate (Staples and Webster, 2008; Mueller and Kamdar, 2011). Furthermore, task interdependence can improve communication and encourage supportive behavior, in which team members consider their coworkers’ interests as well as their own. With a top standard of task dependency, the detrimental effects of knowledge concealing can be mitigated.

The more interconnected the duties, on the other hand, the less probable it is that any single person will possess all of the necessary expertise. Information concealing hinders members of the team from gathering existing expertise from people with the necessary information for increasing intellectual capital for interdependent tasks. Even if one coworker hides information under a high level of task interdependence, the rules of reciprocity and the achievement of shared objectives should motivate his or her colleagues to spread information regardless, resulting in team knowledge transfer (Sargent and Sue-Chan, 2001; Matusik and Heeley, 2005). As a result, under high task interdependence scenarios, the focus on task completion and shared objectives may motivate members of the team to collaborate with one another in exchange relationships, enhancing their capacities to integrate and utilize available knowledge. Therefore, we hypothesized the following.

**H_5_**. Task interdependence moderates the relationship between personal competition and playing dumb.

A following conceptual model (Figure 1) has been formed based on the above literature and hypothesis.

**FIGURE 1:** Theoretical framework. PC, personal competition; PD, playing dumb; TP, team performance.

## Methodology

The present study follows a post-positivist deductive method to check the hypothesis of the study which implies the quantitative research design for the study. A total of five hypotheses have been developed in the present study to check the effect of the independent variable (personal competition) on the dependent variable (team performance). Moreover, the mediating role of the playing dumb variable has been deployed along with the moderation of task interdependence. A survey method using the questionnaire has been used in this study. The questionnaire survey was administered by the authors to avoid any misunderstanding by the respondents; however, the rationality of the data has been made sure by letting the respondents fill the questionnaires without any external pressure. The unit of analysis of the study is individual, i.e., sportsmen who were taken as the population of the study who are involved in sports activities at their school/institute level or play under local sports bodies in China. The data had been collected from the respondents on the basis of convenience sampling as it is cost-effective and data is readily obtained (Dar et al., 2022). The sample size for this study used is 339 sports players.

### Statistical Tool

The structural equation model for the current study had been examined using the software Smart PLS 3.3.3 There are several reasons for using this software. First of all this software helps in examining small data and developing the path models quickly (Avotra et al., 2021). Using Smart PLS, the data is analyzed in two stages. The first stage, measurement model assessment, helps in validating the data through factor loadings, Fornell and Larcker criteria, heterotrait–monotrait (HTMT) ratio, average variance extracted (AVE), and variance inflation factor (VIF). The reliabilities are checked through Cronbach alpha and composite reliability. The hypotheses have been accepted based on the *t*-statistics, sample means, and *p*-values.

#### Measurement

The questionnaire used in this study had been designed on a 5-point Likert scale, consisting of the variables of the study, i.e., personal competition, playing dumb, team performance, and task interdependence. The details for each variable adaptation have been given along with their alpha reliabilities obtained. The minimum threshold mentioned in the literature is 0.7 (Xiaolong et al., 2021; Yingfei et al., 2021). For the data to be reliable, the value of Cronbach’s alpha should be higher than 0.7.

#### Personal Competition

The scale used for the variable personal competition had been adapted from Hernaus et al. (2019). It consisted of four items, showing Cronbach alpha value of (α = 0.883) which is above the minimum threshold for alpha reliability.

#### Playing Dumb

The scale used for the variable playing dumb had been adapted from Connelly et al. (2012). It consisted of four items, showing Cronbach alpha value of (α = 0.917) which is above the minimum threshold mentioned for alpha reliability.

#### Team Performance

The scale used for the variable team performance had been adapted from Bateman et al. (2002). It consisted of eight items in total, but seven items were included in the study because it shows low factor loading (0.314) which doesn’t fall in the acceptable range (Dash and Paul, 2021). After excluding the item TP8 the variable showed the Cronbach alpha value of (α = 0.881) which is above the minimum threshold mentioned for alpha.

#### Task Interdependence

The scale used for the variable task interdependence had been adapted from Sargent et al. (2001). It consisted of four items in total showing Cronbach alpha of (α = 0.888).

### Demographic Details

Results for the demographic profile showed interesting results. The gender-wise participation in the survey was found almost the same. A total of 52% of the participants were male while 48% of the participants were females. The highest number of respondents was found to be between the ages of 15–20, followed by the age category of 21–25 and then the age category 26–30. The age category up to 30 years had been included because usually young adults actively participate in sports activities (Lee, 2020; Marchena-Giráldez et al., 2021). The education category of bachelors (53.6%) and masters (48.3%) showed somewhat the same frequency of the participants. However, 53.7% of the participants had experience in sports activities of less than 1 year; however, it was followed by less than 3 years of experience and the least number of participants had an experience of more than 6 years (see Table 1).

**TABLE 1:** Demographics analysis.

Demographics	Frequency	Percentage
**Gender**		
Male	178	52.50
Female	161	47.49
**Age (years)**		
15–20	161	47.49
21–25	139	41
26–30	39	11.50
**Education**		
Bachelors	175	53.68
Masters	164	48.37
**Experience in sports (years)**		
Less than 1	182	53.68
1–3	98	28.90
4–6	43	12.68
More than 6	16	4.71

*N = 339.*

### Common Method Bias

The biasness of the questionnaire has been checked through the single factor test that was conducted *via* total variance explained (Li and Cao, 2021). The results obtained from this test have been reported in Table 2 (Li and Cao, 2021) have argued that the one-factor test conducted, should show a variance of less than 50% to rule out the possibility of common method bias. The results of the questionnaire used in this study showed 41.5% of the variance, thus indicating the absence of bias.

**TABLE 2:** Total variance explained.

Component	Initial eigenvalues			Extraction sums of squared loadings		
		
	Total	% of variance	Cumulative %	Total	% of variance	Cumulative %
1	7.895	41.551	41.551	7.895	41.551	41.551
2	3.511	18.479	60.030			
3	1.234	6.493	66.523			
4	1.131	5.954	72.476			
5	1.009	5.308	77.785			
6	0.601	3.163	80.948			
7	0.489	2.573	83.521			
8	0.454	2.390	85.911			
9	0.408	2.145	88.056			
10	0.354	1.863	89.920			
11	0.316	1.664	91.583			
12	0.294	1.547	93.130			
13	0.262	1.380	94.511			
14	0.239	1.259	95.769			
15	0.205	1.077	96.846			
16	0.174	0.915	97.761			
17	0.163	0.860	98.621			
18	0.142	0.750	99.371			
19	0.119	0.629	100.000			

*Extraction method: principal component analysis.*

## Data Analysis and Results

### Measurement Model

The measurement model has been represented in Figure 2 of the study. This figure explains the contribution of each predictor variable of the study toward their corresponding dependent variables.

**FIGURE 2:** The output of the measurement model algorithm. PC, personal competition; PD, playing dumb; TP, team performance.

Table 3 shows the factor loadings for every item of the variables of the study, i.e., personal competition, playing dumb, team performance, and task interdependence. The fair acceptance criteria of factor loadings mentioned in the literature are above 0.6 (Nawaz et al., 2020). The factor loading results of the variables have shown significant values except for TP8 showing factor loading of 0.318. Thus, the rest of the analyses have been carried out excluding this item. Furthermore, the values for the outer VIF have also been reported in Table 2. According to Craney and Surles (2007), the values of VIF should be less than 0.5. The present study has ensured the absence of collinearity by indicating the values of VIF less than 0.5. Similarly, the adequate level of AVE has been reported as 0.5 and above (Rani et al., 2018). The present study shows all the values of AVE above 0.5 thus confirming the convergent validity of the study. Similarly, the composite reliability for the variables used in the present study are all above 0.7, thus meeting the acceptance criteria (Bujang et al., 2018).

**TABLE 3:** Measurement model.

Variables	Factor loadings		VIF	Composite reliability	AVE
Personal competition	PC1	0.884	2.984		
	PC2	0.833	2.278	0.919	0.739
	PC3	0.820	1.705		
	PC4	0.900	3.544		
Playing dumb	PD1	0.867	2.365		
	PD2	0.923	4.342	0.942	0.802
	PD3	0.871	2.521		
	PD4	0.919	4.201		
Team performance	TP1	0.758	1.991		
	TP2	0.800	2.798	0.906	0.581
	TP3	0.780	2.387		
	TP4	0.788	1.779		
	TP5	0.759	2.600		
	TP6	0.735	2.357		
	TP7	0.711	2.291		

The discriminant validity in the present study has been found to prevail showing that the variables are different from each other. It has been measured using two mainstream tests of HTMT ratio and the Fornell and Larcker criteria (Afthanorhan et al., 2021). For the data to be discriminately valid the value of the HTMT ratio should be less than 0.85, and for the Fornell and Larcker criteria, the table should show the highest values of each column at the top (Afthanorhan et al., 2021). Table 4 shows the Fornell and Larcker criteria and Table 5 shows the HTMT ratio. The ratios obtained in this study for these two tests are found significant and acceptable to ensure the variables of the present study are different from each other.

**TABLE 4:** Discriminant validity (Fornell and Larcker criteria).

	PC	PD	TP
PC	0.860		
PD	0.733	0.895	
TP	0.421	0.383	0.762

*PC, personal competition; PD, playing dumb; TP, team performance.*

**TABLE 5:** Discriminant validity (HTMT ratio).

	PC	PD	TP
PC			
PD	0.798		
TP	0.462	0.411	

*PC, personal competition; PD, playing dumb; TP, team performance.*

The *r*^2^ values obtained for the present study have been good. According to Franke and Sarstedt (2019) the value of *r*^2^ obtained should be near 0.5. The variable playing dumb has shown the *r*^2^ value of 0.54 while the other variable of team performance has shown the *r*^2^ value of 0.19. Hence, the model can be considered good. Furthermore, the *Q*^2^ value shows the cross-validated redundancy and according to Blomquist et al. (2016) it should be greater than 0. In the present study, the variable playing dumb shows the *Q*^2^ value of 0.40 and team performance shows *Q*^2^ = 0.10 hence, showing a good predictive power of the model. The values for *r*^2^ and *Q*^2^ have been reported in Table 6.

**TABLE 6:** *r*^2^ Values and *Q*^2^ values of the variables.

	*r* ^2^	*Q* ^2^
PD	0.542	0.402
TP	0.190	0.100

*PC, personal competition; PD, playing dumb; TP, team performance.*

### Structural Model

The structural model assessment using 95% corrected bootstrap has been used for the direct paths in the study, has been presented in Figure 3. The acceptance criteria used in this study for the hypothesis are *p*-values, *t*-statistics, and the sample mean.

**FIGURE 3:** Output of structural model (simple model).

The results for the direct and indirect effects have been presented in Tables 7, 8, respectively. The acceptance/rejection had been finalized on the basis of the *p*-values. The hypothesis showing a *p*-value less than 0.05 was accepted, otherwise rejected (Andrade, 2019). The strength of the model is shown by the *f*^2^ values. Its value ranges from 0 to 1 where 0 shows a weak relationship and 1 shows the strength of the relationship (Nawaz et al., 2019). Moreover, the values for inner VIF should be <5, thus indicating the absence of collinearity among variables.

**TABLE 7:** Direct effects.

Paths	H	*O*	*M*	SD	Inner VIF	*f* ^2^	*T*-statistics	*p*-Value	Results
PC → TP	H_1_	0.303	0.307	0.076	2.158	0.053	3.971	0.000	Accepted
PC → PD	H_2_	0.733	0.735	0.034	1.103	1.007	21.483	0.000	Accepted
PD → TP	H_3_	0.161	0.160	0.076	2.158	0.015	2.105	0.036	Accepted

*N = 359.*

***p < 0.001, *p < 0.05.

*H, hypothesis; O, original sample; M, sample mean; SD, standard deviation; VIF, variance inflation factor; PC, personal competition; PD, playing dumb; TP, team performance.*

**TABLE 8:** Indirect effects.

Paths	H	*O*	*M*	SD	*T*-statistics	*p*-Value	Results
PC → PD → TP	H_4_	0.118	0.118	0.058	2.049	0.041	Accepted

*p < 0.05. O, original sample; M, sample mean; SD, standard deviation; PC, personal competition; PD, playing dumb; TP, team performance.

In Table 7, the direct effects of personal competition on team performance and playing dumb have been presented along with the effect of playing dumb on team performance. The first hypothesis of the study indicating the effect of personal competition on team performance has been accepted (*O* = 30.3%, *t*-value = 3.97, *p* < 0.05. Hence, personal competition has been found to have an effect on team performance. However, the *f*^2^ was 0.05, showing a weak effect size (*f*^2^: equal to 0.02 is weak, 0.15 is medium and 0.35 and above shows strong effect sizes (Nakagawa and Cuthill, 2007). The inner value VIF values for all hypotheses were found below 5, thus, ruling out the issues of collinearity. The second hypothesis shows a strong effect of personal competition on playing dumb thus accepting the hypothesis (*O* = 73%, *t*-value = 21.483, *p* < 0.05). The third hypothesis regarding the effect of playing dumb on team performance has also been found significant at *p* < 0.05, and *t*-value more than 1.96 (Winship and Zhuo, 2020).

The indirect effect of personal competition on team performance has been found significant. The fourth hypothesis of the study indicating the mediating role of playing dumb between personal competition and team performance has been found significant at *p* < 0.05 with *t*-statistic > 1.96 and hence, the H4 has been accepted. The results for indirect effects have been reported in Table 8. To check the moderation effect, the measurement model was checked again including the moderating variable, task interdependence in the model to verify the validity and reliabilities of the variables in the presence of a moderator. The results obtained for the measurement model have been reported in Table 9. The results were found to have the validity and reliability of the data retained. Hence, the analysis proceeded to the structural model assessment for moderation. The output figure for moderation analysis has been presented in Figures 3, 4.

**TABLE 9:** Measurement model (with moderation).

Variables	Factor loadings		VIF	Composite reliability	AVE
Personal competition	PC1	0.884	2.984		
	PC2	0.833	2.278	0.919	0.739
	PC3	0.820	1.705		
	PC4	0.900	3.544		
Playing dumb	PD1	0.869	2.365		
	PD2	0.922	4.342	0.942	0.802
	PD3	0.869	2.521		
	PD4	0.919	4.201		
Team performance	TP1	0.759	1.991		
	TP2	0.800	2.798		
	TP3	0.780	2.387	0.906	0.581
	TP4	0.788	1.779		
	TP5	0.759	2.600		
	TP6	0.735	2.357		
	TP7	0.711	2.291		
Task interdependence	TI1	0.859	2.248		
	TI2	0.879	3.099		
	TI3	0.887	2.754	0.922	0.747
	TI4	0.831	2.688		

**TABLE 10:** Moderation effect.

Paths	H	*O*	*M*	SD	*T*-statistics	*p*-Value	Results
PC × TI → PD	H_4_	−0.001	0.006	0.050	0.012	0.991	Rejected

*O, original sample; M, sample mean; SD, standard deviation; PC, personal competition; PD, playing dumb; TP, team performance.*

**FIGURE 4:** Output of structural model (with moderation).

The present study has checked the moderating effect of task interdependence on the relationship between personal competition and playing dumb. However, the results could not support the fifth hypothesis of the study thus rejecting H_5_.

## Discussion

This research focused the competitiveness in terms of personal competition and its impact on team performance. The mediating effects of playing dumb were also evaluated in this. The contingent role of task interdependence among personal competition and playing dumb were also evaluated in the research which contributed to some promising and significant results indicating the fruitfulness of the subject. Personal competition exhibits a high degree of self, success, connection, compassion for others’ well-being, and forgiveness, as well as lower levels of dominant behaviors, violence, and psychopathy. Unlike unhealthy kinds of competition, this attitude represents a healthy and constructive sort of competition (Ryckman and Hamel, 1992; Ryckman et al., 1996, 1997; Collier et al., 2010). Though contextual competitiveness and individual competitiveness are well-known, competition appears to be a communal construct as well. Several, widely obtainable examples of a team’s sustained competitiveness resulting in collective goal attainment may be found in personal anecdotes. The results of this study proved that competition whether it is on a personal level or the team level, it plays an important role in shaping the overall performance of the teams. The contributing factor of competition comes along with cooperation in wider perspectives. Herein the study we just evaluated the competition and personal level which had prominent effects on team performance. The other aspect of personal competition producing negative behaviors in players was also significant, showing that certain behaviors such as knowledge hiding were the outcomes of personal competition. The direct effects of personal competition on playing dumb were promising. According to Connelly et al. (2012), playing dumb is the constituent or type of knowledge hiding in which a person (player in our context) hides the information with the colleagues (team players) for certain reasons. It proved that personal competition could be a negative sort of factor in team performance evaluations.

Once the negative behavior develops due to personal competition, it could lead to disturbed team performance. Our results indicated the same in which playing dumb had an impact on team performance. Similar kind of results was also obtained in some of the previous studies (Winship and Zhuo, 2020). We also studied the dimension of playing dumb as a mediator between personal competition and team performance. Certain studies have also evaluated the mediating role of playing dumb in various perspectives, i.e., interpersonal conflict and psychological strain (Venz and Nesher Shoshan, 2021), territorial feeling, and innovation of employees (Guo et al., 2022), etc. Several researchers have focused on mediating the role of knowledge hiding in different perspectives, i.e., abusive supervision and employee creativity (Jahanzeb et al., 2019). These results also indicated that playing dumb or knowledge hiding could mediate the relationship between personal competition and team performance. although, direct effects were also significant but playing dumb proved to be facilitating the relationship more negatively. In the context of moderating the mediated relationship of personal competition with playing dumb affecting the team performance, we also evaluated the contingent role of task interdependence in our study. When tasks are interdependent from other team members, the relationship between personal competition and knowledge hiding should be less negative (Bachrach et al., 2006; Staples and Webster, 2008). On the one hand, task interdependence as a moderator represents an unproven aspect of the original knowledge-hiding theory (Černe et al., 2014). Thus, the negative effects of knowledge hiding could be mitigated in an environment relating to information exchange and collaboration. Because it highlights the necessity of joint effort and collaboration among team members, task interdependence appears to reflect such a climate (Staples and Webster, 2008; Mueller and Kamdar, 2011). However, the moderating effect of task interdependence between the relationship of personal competition and team performance has not been found to have any impactful contribution toward it.

### Practical Implications

There are a few implications of the study that can help real-world personnel in positively modifying their behavior. First of all, it is the responsibility of the mentor, coach, instructor, or manager to make an atmosphere of healthy competition that does not let the players involved in the playing dumb role of knowledge hiding because it consequently affects the team performance. To improve the team performance, the management must make sure the positive reinforcement of the behaviors thus avoiding the feeling of competition. The management should make the independent groups and teams of the employees/players and hold the performance-based competitions so they would not hide anything from each other thus, minimizing the competition at the personal level.

### Limitations and Future Recommendations

Despite contribution to the theory of competition and performance, the present study has some limitations. First of all, the population this study has taken is the sports players because they are found to have been involved in competition at a personal level relatively more (Hatzigeorgiadis and Biddle, 2002). Therefore, this study should be replicated in the corporate sector to find out the generalization of this study among employees of the organization. Secondly, the mediating mechanism in this theoretical framework needs to be further investigated for example moral disengagement could be the possible mediator for the relationship proposed in this study. Furthermore, the current theoretical framework can be extended by examining the impact of more moderating variables such as social support, organizational climate, workforce diversity, etc.

## Conclusion

Personal competition has been prevailing among colleagues and co-workers ever since to prove better at work than others. Such behaviors have been found to have serious consequences on the overall team performance. In order to examine the impact of personal competition on its related consequent factors, this study has been conducted. This study has examined the effect of personal competition on playing dumb and the team performance among the sports-related personnel in China. The results of the study found that the impact of personal competition is significant on team performance and the playing dumb behavior of knowledge hiding from the teammates. Further, the results showed a significant mediating role of playing dumb between personal competition and team performance. However, the moderating effect of task interdependence between the relationship of personal competition and team performance has not been found to have any impactful contribution toward it. However, the study has certain implications for the real-world corporate sector.

## Data Availability Statement

The original contributions presented in the study are included in the article/supplementary material, further inquiries can be directed to the corresponding author.

## Ethics Statement

The studies involving human participants were reviewed and approved by the Shandong College of Arts, China. The patients/participants provided their written informed consent to participate in this study. The study was conducted in accordance with the Declaration of Helsinki.

## Author Contributions

JL conceived and designed the concept, collected the data, wrote the manuscript, and read and agreed to the published version of the manuscript.

## Conflict of Interest

The author declares that the research was conducted in the absence of any commercial or financial relationships that could be construed as a potential conflict of interest.

## Publisher’s Note

All claims expressed in this article are solely those of the authors and do not necessarily represent those of their affiliated organizations, or those of the publisher, the editors and the reviewers. Any product that may be evaluated in this article, or claim that may be made by its manufacturer, is not guaranteed or endorsed by the publisher.
